# Product Market Competition and Firm Performance: Business Survival Through Innovation and Entrepreneurial Orientation Amid COVID-19 Financial Crisis

**DOI:** 10.3389/fpsyg.2021.790923

**Published:** 2022-03-25

**Authors:** Qiang Liu, Xiaoli Qu, Dake Wang, Jaffar Abbas, Riaqa Mubeen

**Affiliations:** ^1^School of Economics and Management, Liaoning University of Technology, Jinzhou, China; ^2^School of Media and Communication, Shanghai Jiao Tong University (SJTU), Shanghai, China; ^3^Antai College of Economics and Management, Shanghai Jiao Tong University (SJTU), Shanghai, China; ^4^School of Management, Harbin Institute of Technology, Harbin, China

**Keywords:** product market competition, entrepreneurial orientation, innovation, COVID-19, firm performance, Chinese market

## Abstract

The product market competition has become a global challenge for business organizations in the challenging and competitive market environment in the influx of the COVID-19 outbreak. The influence of products competition on organizational performance in developed economies has gained scholars’ attention, and numerous studies explored its impacts on business profitability. The existing studies designate mixed findings between the linkage of CSR practices and Chinese business firms’ healthier performance in emerging economies; however, the current global crisis due to the coronavirus has made product market completion fierce, which ultimately affects business firms’ performance. This study focuses on this logical global challenge, investigates the rationale, and examines product-market completion impact on firms’ performance operating in the Chinese markets. The study collected data from the annual reports of Chinese business organizations with A-share listing and registered with the database of China Stock Markets and Accounting Research (CSMAR). The study employed a Generalized Method of Moment technique and investigated the connection between product market competition and Chinese firm performance. The empirical analysis of this study highlights the conclusion that market competition positively and significantly affected business firms’ performance. This study specified that product market competition play a dynamic and indispensable role in achieving healthier firm performance in the Chinese markets. This study provides valuable insights on practical implications and future research directions for the scholars to draw interesting results with new study models.

## Introduction

The ongoing global economic crisis posed by the COVID-19 infectious disease has developed shocks in both demand and supply sides, which has adversely affected the global economy (Abachi and Iorember, 2017). As a result, this financial crisis has created a demanding and challenging situation for business firms due to slumps in industry and consumer spending (Abbas et al., 2021). It has created disruptions in economic activities and supply chains, which ultimately affected firms’ performance. The coronavirus outbreak has deep integration with global economies. It has affected enterprises and corporations’ business activities globally (Su et al., 2021b). A study specified that the progress of Vietnam GDP was much slower and showed only 3.8% growth and further expected to remain around 3–4% compared to 6.5%, which is the lowest in the last 10 years. Similarly, this crisis has influenced the economies of all the countries and posed severe challenges and a turbulent industry environment for business firms. The occurrence of emergencies and global economic crises adversely influences society’s particular aspects and business firms’ strategic innovation (Yang et al., 2020; Huang et al., 2021; Zhang and Zhu, 2021). The global health crisis and public emergencies increase raw materials procurement costs, restrict employees from joining the workplace, create challenges for business entities to resume work schedules, and ultimately firms struggle to survive in the crisis (Gugler et al., 2020; Howell, 2020; Chebolu-Subramanian and Sundarraj, 2021).

Restriction during the pandemic caused production shutdowns, shortage of raw materials supply to produce final goods, delays in sales of products and services, disruptions in economic activities, and supply chains posed severe challenges to business firms in the emergence caused by COVID-19 pandemic (Rahman et al., 2021; Saifuzzaman et al., 2021). It has adversely affected business enterprises cash flows and caused a liquidity crisis (Gubareva, 2020; Farzami et al., 2021; Zaremba et al., 2021). The outbreak of epidemics and pandemics create global health challenges and economic crisis (Yoosefi Lebni et al., 2020, 2021) and negatively affect employees’ emotions (Zhou et al., 2022), which results in harmful effect on innovative employees’ behavior (Moradi et al., 2020; Azadi et al., 2021; Lebni et al., 2021; Su et al., 2021d). Employees negative emotions creates hurdle to improve firm innovation, which affect product competition (Zhang et al., 2017). Educating employees on how to cope with the pandemic can reduce their mental stress, which will improve employees’ productivity for firms (Maqsood et al., 2021; Rahman et al., 2021). The pandemic has posed psychological and physical violence, which has influenced on mental wellbeing. Social media technology typically plays a positive role in providing timely, precise and valuable health-related information to business firms and employees (Abachi and Iorember, 2017; Lebni et al., 2020; Nasifoglu Elidemir et al., 2020; NeJhaddadgar et al., 2020b; Ge et al., 2021). Business organizations providing social support to their employees create a peaceful working environment and encourage them to deliver maximum productivity to improve firm performance. While the coronavirus outbreak posed indelible damage to the business firms, the COVID-19 has also created opportunities and new pathways to grab the market share through innovation and competitive products. It leads researchers to conduct further detailed studies to enrich innovation theories’ implications to guide business firms to prepare business strategies to respond to the economic crisis and survive in the industry. Consequently, it is theoretical way and practical approach to explore the COVID-19 impacts on the innovation process, which helps achieve better firm performance.

Many organizations consider corporate competitive strategies to increase likely competitive advantages (Hitt et al., 1996), CSR activities improve firm performance (Hussain et al., 2017), increase business firms market share (Franko, 1989), and enhanced organizations performance (Giroud and Mueller, 2011). Because competitive strategies are used as an important tool to achieve firm objectives. Many scholars have paid attention since long and showed interest in corporate strategies, and focused on examining the link between firms products competition and firm performance (Raith, 2003; Pant and Pattanayak, 2010; Sheikh, 2018; Javeed et al., 2020). Existing studies revealed mixed findings on this relationship. For instances, Raith (2003), Pant and Pattanayak (2010), and Sheikh (2018) identified that products competition at marketplace positively improves business organizations performance. On the other side, another study reported that products competition is keen and it creates a competitive setting for businesses and corporations, which leads low pricing power and thus low profits (Javeed et al., 2020). The consequences of the impact differ greatly due to the different data, times periods, and different performance measurement. Consequently, academics recommend that for analyzing the real impact of products market competitiveness on better performance needs further investigations (Guney et al., 2011; Sheikh, 2018). It is due to the COVID-19 outbreak, which has developed profound adverse effects on the world economy (Crick and Crick, 2020). Therefore, based on these rational and logical claims and the existence of this gap, this study examined the role of companies’ products competition at market toward better firm performance.

This research is primarily engrossed in exploring firms’ product(s) competition and its influence on firm performance in the context of China. Using the GMM model, the study findings offer helpful/valuable insights and specified that Chinese firm products’ competitiveness at the marketplace developed a positive link to better performance. The study results designated that the chosen variable has positively influenced better performance, which confirmed that companies’ product competitiveness enhances firms’ profitability. In brief, this study has provided valuable and critical contributions to the literature related to companies’ products and services competitiveness. In the first phase, product competitiveness helps achieve better profits and enhanced performance. This present research model contributes to testing product competition in the marketplace and its influence on a firm’s profitability and healthier performance. In the second step, the study has employed the GMM model to investigate the chosen framework and test the endogeneity issues in this present research. The third phase promotes companies’ product competition in the Chinese business industry and other developing economies. This study arrangement follows the organization as follows. The study overviewed the role of business firms’ innovativeness, resources in hands, business networks, and dynamic capabilities that affect to produce the best products to compete in the business competition, which ultimately enhances firm performance. These influential factors help firms to survive in the time of emergencies and global crises. In the second phase, the study describes the methodology section for the selected exploratory research. In the third step, this study has elaborated the compelling findings and factors that affect firm performance at all times, including the financial crisis. In the final section, the study concludes the discussion with suggestions and limitations.

## Literature Review

Eggers (2020) conducted a study and examined 69 research articles that explored the business companies’ behaviors in past emergencies/crackdowns, and the findings proposed possible helpful pathways to overcome economic crises (Eggers, 2020). The study identified that most former researchers emphasized managing economic indicators, such as profitability, debt ratio, action plan, affecting liquidity, creditworthiness, dynamic capabilities, products competition in the market, and financial safety amid an economic recession or downturn (Lisboa, 2017; Duarte et al., 2018; Brown and Lee, 2019). However, these earlier researches have not emphasized possible pathways to manage and overcome financial distress and crisis. These studies had primarily ignored and did not focus on exploring the relationship between business firms’ coping strategies and healthier financial performance during emergencies. Past studies recognized that the assets of the business firms, corporations, and SMEs are critical elements that companies will remain in the business industry during economic crises and emergencies. Another study examined firms strategies in the emergencies and described that companies, which followed entrepreneurial orientation, had shown more incredible innovation, effectiveness, and risk-taking (Soininen et al., 2012). It was a practical action for the business firms to remain in the business industry in the middle and after a crisis. Some studies identified that the emergencies and economic crises positively influenced the business firms for their development and proactive movements, improving firms’ corporate performance during emergency times.

This study contributes to firm performance literature. This study has provided valuable insight for the business owners, CEOs, decision-makers, and business managers on coping with the economic crisis and financial distress posed by the COVID-19 outbreak. The study explains that business organizations’ behavior is critical in emergencies. Business firms’ resources, entrepreneurial factors, dynamic capabilities, innovativeness, and coping strategies to combat the adverse effects play indispensable roles in surviving in a crisis. The governments can play an essential part in providing support for SMEs to keep them active to combat the COVID-19 impacts during the crisis. Thus, SMEs are the engine of the economy and create economic activities on a large scale. The combined global efforts are helpful to fight against the COVID-19 adverse effects on business organizations. The business managers’ point of view is critical, as their concern is to reduce the COVID-19 spillover effects when opting for coping strategies during the crisis. The existing financial global challenge posed by the pandemic (COVID-19) has created an economic crisis ranging from weak industrial output to severe market competition across the globe. The pandemic has also affected environmental sustainability adversely and disrupted economic activities worldwide (Goshit and Iorember, 2020; Iorember et al., 2020, 2021; Jelilov et al., 2020; Usman et al., 2020). Recent researches have shown that the response of monetary aggregated necessary to support industrial performance within the pandemic period is weak relative to the period before the pandemic (Abachi and Iorember, 2017; Iorember et al., 2019; Usman et al., 2019; Dabwor et al., 2020; Goshit et al., 2020).

Corporate firms’ competitiveness is vital in determining the organizations corporate level strategies. Organizations incorporate these useful strategies to attain competitive benefits (Hitt et al., 1996; Mubeen et al., 2016). Organization’s strategies help achieve market share expansions (Franko, 1989), higher profitability and better firm performance (Giroud and Mueller, 2011). Companies’ product competitiveness in the industry help in attaining business goals (Giroud and Mueller, 2010; Tian and Twite, 2011; Ko et al., 2016). Business managers’ focus on achieving better financial performance and it ties up to achieve better performance, which ultimately enhances firms’ profitability. Earlier research identified that product competition is a helpful approach for firms’ managers, motivating them to increase income for the stakeholders. It helps reduce the expense of agencies and leads to higher profitability for business firms (Ammann et al., 2013). Past research examined 670 UK-based business firms from 1972 to 1986 and recognized that products competitive nature having more competitor firms, or lower rents helped various firms profitability and better performance. The literature has evidenced and stated that competition boosts productivity and impact positively on firm performance (Nickell, 1996; Mnasri and Ellouze, 2015). The existing research literature has concluded that entrepreneurial resources are active agents in mitigating the COVID-19 crisis adverse effects on business firms (Scheidgen et al., 2021). However, the literature has designated the mixed results related to firms’ competitive products and their influence on better profitability. Some research has shown that product competitiveness provides a positive impact, while some studies identify a negative relation to better firm performance. The findings of empirical studies indicated that product competition leads to achieving better performance and higher profits because firms’ competitiveness resolves agency conflicts between stakeholders, owners, and managers, which results in better profitability of the firms (Raith, 2003; Ruiz-Porras and Lopez-Mateo, 2011; Mubeen et al., 2016).

Concerning the challenging financial crisis, business firms have modified their business model by shifting the cooperation (competition) between competing organizations. Some research from the emerging markets identified that product competition is helpful and creates a positive impact on business organizations’ healthier performance. The present study’s findings are consistent with the literature and proved that product competition enhances firms’ profitability, better performance, and positively influencing higher sales (Javeed et al., 2020; Mubeen et al., 2020). Based on the arguments above, the literature empirically recognized that product competition positively influences business firms’ performance with higher profitability. The study proposes and hypothesizes the following statement.

**Hypothesis 1(H1):** Product market competition, innovation and entrepreneurial orientation positively influence firm performance.

## Methodology/Materials

### Research on Panel Dataset

This study primarily analyzed the association between product competition and business firms’ performance. The study collected panel data (2016–2020) from the annual reports of Chinese business organizations with A-share listing and registered with China Stock Markets and Accounting Research (CSMAR) database. The study employed a Generalized Method of Moment technique and investigated the connection between Chinese firms’ product competition in the market and its influence on the firms’ performance. The GMM regression analysis requires at least 3 years of panel data from the companies with consecutive observations. This study has used the GMM model instead of the panel-data regression approach due to the following reasons. In the regression model, when there is a correlation between the error terms, the variables face endogeneity problems. Similarly, these problems may also result from automatic regression or missing variables, measurement errors, and autocorrelation errors (Singh et al., 2018). According to the econometrics rules, if there is just one endogenous variable in the research framework/model, then an appropriate technique is helpful to solve the endogenous problem (Javeed et al., 2020).

### Variables Definition

#### Business Firm’s Product Competition

Product market competition is the key independent variable in this present proposed study model. Previous studies have indicated that the HHI technique (Herfindahl-Hirschman Index) is the best suitable measurement approach among the other available methods to assess market competition and product performance. Researchers usually employ the HHI-score method to evaluate and analyze market concentration. Scholars use HHI approach in determining market competitiveness. HHI method stems from the realism that helps measure simple market competition scenarios. It does not support measuring various markets volatility and complexities (Zou et al., 2015). HHI-score helps scholars to calculate and determine the size of the organizations concerning the business industry. The HHI-score is an indicator to specify market competition level among business firms. HHI is an economic concept, and scholars broadly use it in antitrust, competition law, and technology management (Liston-Heyes and Pilkington, 2004). The significant advantage of the HHI-score linkage to the business industry helps measure the concentration ratio, which allocates more weightage to large business firms. Other considerable benefits of HHI include its easy and straightforward measurement method of market concentration. It needs small data for the market competition calculation (Kvalseth, 2018). HHI-score calculates the market concentration of the top 50 business firms operating in a specific industry to determine whether that particular business industry is competitive or working close to a monopoly. It helps determine the concentration ratio of the number of business firms that produce or market a specific product or a series of products accompanied by the relative distribution channels of market share for each firm’s sales volume in the specific industry. According to economists, market concentration share is a critical determinant that indicates market completion violability and choice of consumers (Lee et al., 2020). Following the existing researches (Michaelides et al., 2019; Javeed et al., 2020) this present study has measured and evaluated market competition and applied the sum of squared based on firm’s market share operating in the industry considering firm’s total sales volume in the specific Chinese business industry (Mubeen et al., 2020).

#### Firm Performance

The present study has designed a framework/model based on the literature support and chosen firm performance as its dependent variable, whereas, firms’ product competition is the independent variable. The existing literature has not documented specific measurements in calculating the performance of business firms. However, the literature has shown that various methods are helpful to measure the organizational performance of the business entities, such as return on assets (ROA), return on investment (ROI), return on equity (ROE), Tobin Q and dividends payable (Javeed et al., 2020). However, in this paper, we use ROA and ROE measures as our performance measurements. Hutchinson and Gul (2004) and Javeed et al. (2020) reported that accounting-based measurement methods are most suitable for corporate governance research literature because these measurement methods can easily track the ability to manage the value of the company.

The proposed research framework shows this relationship. Scholars measure the profitability of business firms by using the return of equity mechanism. ROE helps calculate a firm’s viability in relation to its equity. Experts estimate the equity of a firm’s shareholders by taking all firm’s assets and then subtract all outstanding liabilities. ROE is also a determinant of return on assets minus the firm’s liabilities. Return on firm’s equity (ROE) shows that how well is the profit in dollars from the investment of each dollar for the shareholders’ equity. ROE metric specifies that how good business firms utilize their equities to generate attractive profits for the shareholders (Altı and Sulaeman, 2012; Bathia et al., 2020). ROE helps measure how well business firms are performing in the same business industry. ROE is a measurement tool to know about the ability of management to generate income from a firm’s equity in hand. Experts consider a return of 15–10% as a good income for investors (Bunea et al., 2019; Hibbert et al., 2020).

The existing literature reported that accounting-based measures are the best practices, and using corporate governance empirical studies results are helpful (Bunea et al., 2019). In this practice, the management’s ability linked to the value of business firms is easily to understand and traceable with the measures of corporate governance practices (Mubeen et al., 2020). Consequently, this present study has incorporated ROE, stating return on firms’ equity as a performance measure by following the previous studies exploring corporate governance effects on selected firms’ performance (FP), which is the dependent variable here in this model. This study measured ROE as business organizations operating profits ratios to shareholder equity (Bhagat and Bolton, 2008; Javeed et al., 2020). Besides, scholars broadly employ ROE to evaluate and judge firms’ performance measures in corporate governance research studies because researchers primarily investigate ROE in corporate governance studies (Bathia et al., 2020; Andersen et al., 2021). According to the stakeholder viewpoint, ROE is the best way to test a firm’s business performance (Brown and Caylor, 2009).

#### Control Variables in the Proposed Model

This study has employed some control variables, which is helpful to receive suitable study results. The control variables include the organization’s capital structure, growth, firm size, and asset tangibility. Sales growth of the business organization (Growth) is the proxy related to firms growth opportunities, and the study calculated it by recording changes in firms sales revenue (King and Santor, 2008). Besides, the study measured firms’ assets tangibility determining it ratio of the plant equipment and firms overall revenue. The literature evidenced that corporate finance researches mostly take firm size as a vital study variable. This model also assessed the firm size and took it as a log of firms sales volume (Mahmood et al., 2019). This study calculated business organization’s capital structure, which determines debt-to-equity ratio, and delivered interesting and consistent findings with the previous research results (Mubeen et al., 2016, 2020; Mahmood et al., 2019).

#### Empirical Examination

This current study has gathered panel data based on the annual financial statement and equity details from Chinese firms, rated with A-share star and registered with China Stock Markets and Accounting Research (CSMAR) database to draw the results. The present study has taken A-rated shares business firms by following the previous studies (Zhao et al., 2018; Guo et al., 2020). This study employed random sampling techniques and selected the required data by following the previous literatures (Zhao et al., 2018; Guo et al., 2020). In the next stage, the study applied a Generalized Method of Moment approach and examined the link between product competition in the market and Chinese firms’ profitability and enhanced results. The empirical analysis of this study indicated that market competition positively affect business performance. This study specified that product competition play a dynamic and indispensable role in achieving healthier firm performance in the Chinese markets. The empirical analysis of the regression model generally reports endogeneity issues, which generates unreliable and biased results (Akram et al., 2017; Khan et al., 2017; Javeed et al., 2020). Concerning the rule of econometric, if the study model contains just one variable with endogenous problems, then the model needs to incorporate suitable passable methods to deal with the issues of endogeneity (Mubeen et al., 2020). The formation of the panel dataset places limitations on the applicability of the OLS method (Ordinary-Least Square). The OLS model leads to biased estimation in the results due to unobserved heterogeneity (Zou et al., 2015; Javeed et al., 2020). This study employed the GMM and tested model’s heteroscedasticity and autocorrelation to deal with endogeneity issues.

## Results and Findings

### The Chosen Model’s Descriptive Statistics

This study has presented descriptive analysis as indicated in Table 1 that demonstrates the chosen model of the study. The study model has incorporated the Chinese business firms’ performance as DV (dependent variable) and product competition as IV (independent variable). The literature exhibited that various scholars display descriptive statistics in the empirical results as descriptive analysis provides statistics summary and summarizes the features of the received panel dataset (Illowsky and Dean, 2017; Aman et al., 2019b; Aqeel et al., 2020). Table 1 exhibits the summary information of the descriptive analysis of the study model. The average value of ROE (equity value) of the model is 0.2471; the Std. value is 0.726, and the mean score of firm product competitiveness (HHI) is 0.851, along with a Std. score of 0.389, respectively. The capital structure has exhibited a mean score of0.0715, along with the Std. score of 0.088. The mean score of the firm size is 9.42, Std. score 0.745 and assets tangibility average value remained 0.278 along with Std. value 0.165. The Chinese business firms’ growth exhibited an average value of 0.151, Std. value 0.111. See Table 1, which exhibits the summary information of descriptive analysis, demonstrating mean scores, Std. value, minimum and maximum scores.

**TABLE 1:** It exhibits mean scores, Std. value, minimum and maximum outcomes.

Variables	Observations	Mean	Std.	Min	Max
Return on equity (ROE)	1,668	0.2471	0.726	–6.02	4.74
Market competition	1,668	0.815	0.389	0	1
Capital structure	1,668	0.0715	0.088	0	0.503
Size	1,668	9.42	0.745	0.00	11.82
Asset tangibility	1,668	0.278	0.165	0	0.835
Growth	1,668	0.151	0.111	0.0005	0.740

*ROE, Return on firm’s equity; Std, Standard deviation.*

### Correlation Matrix

This present study model observed that most of the selected independent variables reported correlational relations below 20%. It designated that multicollinearity had not appeared to report any significant issues for analyzing the proposed study model in absolute terms. This study recognized that correlational linkage to most variables remained lower than almost 20% in absolute terms. The empirical analysis of the panel dataset in this model revealed that the chosen variables correlations remained below 20%, which exhibited that the model has no issues of multicollinearity (Gupta et al., 2018; Mamirkulova et al., 2020). See Table 2 that explains the correlations between the chosen variable in this model.

**TABLE 2:** Correlation matrix of the study model.

Factors	ROE	HHI	Firm size	Liquidity	Capital structure	Asset tangibility
ROE	1					
HHI	–0.00801	1				
SIZE	0.270***	–0.00708	1			
Growth	0.245***	0.0185	–0.0167	1		
Capital structure	–0.154***	–0.00652	0.196***	–0.226***	1	
Asset tangibility	–0.236***	–0.00495	0.205***	–0.379***	0.291***	1

Significance levels @ (i) *p < 0.1, (ii) ***p < 0.05, (iii) ***p < 0.01, ROE explains “return on firm’s equity” and HHI describes Herfindahl-Hirschman Index.

### Regression Analysis

This empirical study hypothesized that Chinese organizations’ entrepreneurial and innovation strategies and product competitiveness helps business firms to increase profitability and business growth. The research proposed the hypothesis that there exist the significant positive link between firm’s product competition in the market and better business firm’s performance. Table 3 displays the empirical outcome of the model and reveals dependent (firm performance) and independent (product competition) variables results, and confirmed the positive relationship between the chosen variables. The findings exhibited that product competition positively influences firms’ performance and increases profitability. The HHI coefficient score remained 1.86 at a 1% significance level, along with ROE (return on firm’s equity). As indicated in Table 3, the study results confirmed the relationship of the hypothesized statement that product completion strengthens firm performance in a positive direction. The study findings of this model are in line with the past research results (Pant and Pattanayak, 2010; Ammann et al., 2013; Li et al., 2018). Another previous research identified similar results that firms’ product competitiveness helps increase sales and profitability and confirms that product competition positively influences business organizations’ better performance (Javeed et al., 2020). Besides, business organizations focusing on more incredible market completion approach improve their corporate financial performance as they build a good corporate stature in the industry and society (Porter and Van der Linde, 1995). The developing economies’ business firms have paid more attention to build their positive corporate image in the industry and tried to remain unique. The firm’s management understands that creating a good image will help increase higher sales and better profits. The study findings provide insights for decision-makers, entrepreneurs’ networks, business owners, managers, and policymakers to prepare suitable strategies to create higher sales to remain competitive in the business industry. Consequently, competition motivates business organizations from the developing economies to stay competitive by launching entrepreneurial and innovation strategies to offer innovative products to capitalize on the benefits as the first mover to gain maximum profits from the industry. The competitive business environment builds pressure on relevant business managers to achieve their targets with dedication and full of motivation to maximize the firm’s profitability (Raith, 2003; Li and Li, 2018; Javeed et al., 2020; Yung and Nguyen, 2020; Carter et al., 2021). The competitive business environment encourages managers to perform well, and fiercely competitive markets do not allow managers to utilize the firm’s resources for personal usage (Januszewski et al., 2002; Allee et al., 2021; Won Henny Jung and Subramanian, 2021). Table 3 shows ROE here.

**TABLE 3:** It exhibits product competition and its influence on Chinese firm performance.

Variables	ROE
HHI	1.865 *** (0.347)
Capital structure	–3.71*** (0.909)
Size	2.57 *** (0.354)
Asset tangibility	–2.80*** (0.615)
Growth	–0.670*** (0.708)
Constant	–24.37*** (3.55)
AR(1)	–2.35
AR(2)	0.29
Sargan test	157.12
Observation	1,668

Significance levels @ (i) *p < 0.1, (ii) ***p < 0.05, (iii) ***p < 0.01, ROE shows, “Return on firm’s equity.”

## Discussion

This present study primarily emphasized reconnoitering the COVID-19 outbreak adversative business effects on firm performance. This study investigates the research question concerning the challenging environment in the industry due to the COVID-19 pandemic. This research explores how business firms achieve better business profitability and better performance in the competitive industry environment amid pandemic crisis. The present study examined firms’ innovativeness, available resources, competence, entrepreneurial networks, and dynamic capabilities, and social media use (Abbas et al., 2019; Crick and Crick, 2020), which influence producing good products to survive in the competitive business environment. Social media technology in the advent of the pandemic (COVID-19) has helped business organizations to seek the latest information about the crisis to take protective measures for the safety of their personnel (Abbas et al., 2021). The workforce and management’s mental wellbeing is essential to achieve better firm performance. The competitive behavior of business firms keeps them vibrant and active that ultimately improves firm performance (Pantano et al., 2020). The COVID-19 economic crisis posed challenges as well as provided marketing innovation and digitalization opportunities to capitalize on business openings with competitive products to survive in the crisis (Seetharaman, 2020; Wang et al., 2020).

Business firms’ have adopted new pathways to survive in the crisis posed by the COVID-19 pandemic. Organizations strive for maintaining the sustainability through competitive activities. The competitive firms allow business activities and provide opportunities to meet with demands of the customers and business environment requirements, which have resulted in before the crisis and increased during this era of the COVID-19, such as additional services and digital solutions (Ilinova et al., 2021). The influential elements help firms in surviving in the competitive business during the economic crisis (He and Harris, 2020). The tourism firms practicing CSR activities during the COVID-19 pandemic have received good response from the customers (Aman et al., 2019a; Mamirkulova et al., 2020). Firms contributing to social good and society remain in the competitive environment, which improves business performance.

Scholars have debated the business firms’ behaviors during the economic crisis challenges and identified that firms’ dynamic competencies, entrepreneurial resources are critical. The real estate firms have reported mixed results in the pandemic crisis as market value and rental prices revealed different results (Hussain et al., 2019, 2021). These factors determine probability and business growth in the turbulent and challenging time of emergency (Mubeen et al., 2020; Raza Abbasi et al., 2021). These determining factors help survive business firms during odd times, and firms’ entrepreneurial resources help them stay in the economic crisis. Business firms with rich resources, such as dynamic capabilities, entrepreneurial orientation with more proactive, innovative, and willing behaviors to face business risk, attain greater chances to survive through and after the economic crisis (Soininen et al., 2012; Abbasi et al., 2021a). Past studies have designated that business firms’ innovativeness, business networks, coping strategies implications and proactive moves positively influence business performance (Meutia et al., 2018; Dias et al., 2021). The demand for renewable energy has been increased to manage environmental issues (Abbasi et al., 2021b).

The pandemic (COVID-19) appearance has posed unprecedented and extreme business cases to learn and examine business activities’ adverse and spillover impacts on business firms worldwide (Akhtar et al., 2019a,b, 2020; Siddiqi et al., 2020; Dias et al., 2021). The pandemic has massively influenced tourism and hospitality business firms (Siddiqi et al., 2019; Akhtar et al., 2021a,b; Islam et al., 2021b). The advent of the pandemic COVID-19 has resulted a steep decline in business activities of hospitality business firms (Anser et al., 2020; Islam et al., 2021a). The literature has overlooked to explore the combined impact of the interaction between business organization’s economic growth in the time of crisis and firms entrepreneurial resources and coping strategies selection in the context of social and financial crises. This study aims to identify this unique context, address the identified research gap. It explores interrelationships between firms’ coping strategies in crisis, resources in hand, innovativeness, and entrepreneurial networks. Based on the discussed research gap, this study investigates the factors that influence firm performance during a time of crisis or emergency and how product market competition affects organizations’ business performance.

An earlier study explored the adverse influences of the COVID-19 outbreak on business firms’ innovativeness, and findings indicated that Chinese listed firms’ innovation input has increased in the emergence of the pandemic. However, innovation input improvements do not mean the implementation of improvements in business organizations (Han and Qian, 2020). Therefore, this study objectively focuses on exploring the product competiveness and firms’ innovativeness effects to achieve healthier performance at all times in general and during the crises in particular (Anjum et al., 2017; IJERPH Editorial Office, 2021; Local Burden of Disease HIV Collaborators, 2021). This study sequence follows the organization as follows. The study overviewed the role of business firms’ innovativeness, resources in hands, business networks, and dynamic capabilities that affect to produce the best products to compete in the business competition, which ultimately enhances firm performance. These influential factors help firms to survive in the time of emergencies and global crises. In the second phase, the study describes the methodology section for the selected exploratory research. In the third step, this study has elaborated the compelling findings and factors that affect firm performance at all times, including the financial crisis. In the final section, the study concludes the discussion with suggestions and limitations.

Many scholars have emphasize investigating direct relationships between product competition and its impact on firm performance. Some of them provides positive relationships (Ruiz-Porras and Lopez-Mateo, 2011; Van Reenen, 2011; Javeed et al., 2020), while others negative or U shape (Januszewski et al., 2002; Bloom et al., 2010; Ko et al., 2016). These studies did not clarify how product market competition can be associated with firm performance positively, negatively, or neutrally. The exiting literature documented many studies that suggested exploring the effects of products competition in the turbulent business environment and how product completion influences firms’ growth (Guney et al., 2011; Sheikh, 2018). Therefore, based on these rational reasons and the existence of this gap, this present model examined the role of market competition on Chinese business firms’ performance. The study has employed the GMM model, and found that product competition in the market leads to better profitability and healthier performance of enterprises and confirmed the positive and significant linkage. The outcomes of this study shows that firms competition builds pressures on business managers to perform well assigned tasks with full devotion to realize profitability of the business firm (Raith, 2003). Based on the consequences of this research, this study provides suitable suggestions for the management, policymakers, stockholders, and owners of developed world industries, along with firms operating in developing economies (Li et al., 2022). Since, vaccines is not available equally across the world, safety measures and employees’ health security is the most important factor (Su et al., 2020, 2021a,2021c; Aman et al., 2021). The emergence of the ongoing pandemic has raised concerns about health priorities for everyone, and social media use has increased to seek health-related information (Pouresmaeil et al., 2019; Abbas, 2020; Fattahi et al., 2020; NeJhaddadgar et al., 2020a; Sarfraz et al., 2021; Toqeer et al., 2021). It provides useful information to improve firm profits at all times, particularly in the emergence of the economic crisis. The study results are helpful for business firms for attracting stakeholders, and other investors to contribute in a competitive environment. This study recommends future research directions to examine different variables that impact firm performance during the crisis, for instance, the role of governance structure, financing configuration, enterprise pattern, business networks, entrepreneurial orientation, competence, innovation, and corporate governance. The prospective studies can investigate the linkage of these factors with product market competition to achieve better firm performance by choosing various firms sectors.

## Conclusion

Scholars have paid attention to discover the direct linkage between product’s market competitiveness and business firm performance; however, the literature showed mixed results. Previous research has not described how product market competition negatively, neutrally, or positively affects organizational performance. Past literature specified that some studies had identified a positive links between product’s competition and improved firm performance. The present research model’s findings are consistent with this argument and designated product competition positive influences on firm performance. This present model recommends exploring the real influence of product competition through mediating and moderating variables on firm performance would produce interesting results. This study incorporated the GMM model technique and recognized that product’s competition positively influences firm performance, confirming the proposed hypothesis of this study. The present article provides a helpful contribution to the literature on business organizations’ performance. This study provides valuable insights for business owners, CEOs, decision-makers, and business managers on dealing with the economic crisis and financial disaster caused by the COVID-19 outbreak.

This study shows that the behavior of business organizations is critical in emergencies and economic crisis. Firms’ resources, entrepreneurial factors, dynamic abilities, innovation, and practical strategies help combat the negative impacts of the pandemic in crisis survival. Governments can play a crucial role in supporting SMEs to keep them active in combating the adverse influence of the pandemic (COVID-19) during the financial crisis. Enterprises’ play an indispensable role to boost business activities. Similarly, SMEs provide a major portion to GDP and they are the engine of the economy in creating large-scale economic activities. Joint global efforts help combat the negative COVID-19 effects on business organizations worldwide. The point of view of business managers is critical, as their interest is to reduce the indirect effects of COVID-19 when choosing crisis confrontation strategies. This present research primarily aimed to explore business firms’ product market competitive situation to attain better performance. Past literature remained unnoticed to examine the collective influence of interaction between firms’ performance and organizational, entrepreneurial orientation and coping strategies during the economic crisis. This research focused on addressing this literature gap. The study investigated interlinked associations between coping strategies, innovativeness, and entrepreneurial orientation in the arrival of the pandemic COVID-19 that caused disruptions and global economic crisis (Mubeen et al., 2021a,b; Aman et al., 2022; Mamirkulova et al., 2022; Zhou et al., 2022). Based on the above debate, the study examined compelling factors that influence firm performance.

### Limitations

This study inherits some limitations like any empirical research study. This study has analyzed the secondary data on annual reports of the A-share listed Chinese business organizations. The Chinese enterprises follow unique state controlled business environment, which is different from other regions across the world. China is the global export leader and the world’s second largest economy. Chinese firms operate under unique capital structure and state monitored corporate sector. Thus, results generalizability of this study does not apply other global economies. Conversely, the literature documented relatively just few studies that explored multiple aspects effects on firm performance. Alternatively, this study’s limitations are helpful, provide the potential for future research, and may help understand the link between competitive products and firm performance. Future research studies can investigate other factors, such as governance structure, corporate governance, and financing allocation through different research methodologies such as cross-sectional design or mixed methods. Future studies can explore more data sets or sectors to understand the relationship between competition in the product market competition and company performance.

## Data Availability Statement

The original contributions presented in the study are included in the article/supplementary material, further inquiries can be directed to the corresponding author/s.

## Author Contributions

RM edited the revised manuscript and contributed to the study design, analysis, literature, discussion, and conclusion. JA conceptualized the idea, contributed to the study design, completed the entire article, including introduction, literature, discussion, conclusion, and edited the original manuscript before submission. DW reviewed and approved the final edited version, and supervised this research. All authors contributed to the article and approved the submitted version.

## Conflict of Interest

The authors declare that the research was conducted in the absence of any commercial or financial relationships that could be construed as a potential conflict of interest.

## Publisher’s Note

All claims expressed in this article are solely those of the authors and do not necessarily represent those of their affiliated organizations, or those of the publisher, the editors and the reviewers. Any product that may be evaluated in this article, or claim that may be made by its manufacturer, is not guaranteed or endorsed by the publisher.

## References

[B1] AbachiP.IoremberP. T. (2017). Macroeconomic and household welfare impact of increase in minimum wage in Nigeria: A computable general equilibrium model. *Am. J. Econ.* 7 249–258.

[B2] AbbasJ. (2020). The role of interventions to manage and reduce Covid-19 mortality rate of the COVID-19 patients worldwide. *Found. Univ. J. Psychol.* 4 33–36.

[B3] AbbasJ.AmanJ.NurunnabiM.BanoS. (2019). The impact of social media on learning behavior for sustainable education: evidence of students from selected universities in Pakistan. *Sustainability* 11:1683. 10.3390/su11061683

[B4] AbbasJ.WangD.SuZ.ZiapourA. (2021). The role of social media in the advent of COVID-19 pandemic: crisis management, mental health challenges and implications. *Risk Manag. Healthc. Policy Vol.* 14 1917–1932. 10.2147/rmhp.S284313 34012304PMC8126999

[B5] AbbasiK. R.AbbasJ.TufailM. (2021a). Revisiting electricity consumption, price, and real GDP: a modified sectoral level analysis from Pakistan. *Energy Policy* 149:112087. 10.1016/j.enpol.2020.112087

[B6] AbbasiK. R.AdedoyinF. F.AbbasJ.HussainK. (2021b). The impact of energy depletion and renewable energy on CO2 emissions in Thailand: fresh evidence from the novel dynamic ARDL simulation. *Renew. Energy* 180 1439–1450. 10.1016/j.renene.2021.08.078

[B7] AkhtarN.AkhtarM. N.UsmanM.AliM.SiddiqiU. I. (2020). COVID-19 restrictions and consumers’ psychological reactance toward offline shopping freedom restoration. *Serv. Ind. J.* 40 891–913. 10.1080/02642069.2020.1790535

[B8] AkhtarN.ChenX.SiddiqiU. I.ZengG.IslamT. (2021a). Language constraints in hotel attributes and consumers’ offendedness associated with behavioral intentions. *Asia Pac. J. Market. Logist.* 33 1–14. 10.1108/apjml-05-2020-0375

[B9] AkhtarN.SiddiqiU. I.AhmadW.UsmanM.ChenX.IslamT. (2021b). Effects of service encounter barriers on situational abnormality and consumers’ behavioral intentions at food and beverage restaurants. *Asia Pac. J. Market. Logist.* 33 1513–1534. 10.1108/APJML-03-2020-0192

[B10] AkhtarN.SunJ.AkhtarM. N.ChenJ. (2019a). How attitude ambivalence from conflicting online hotel reviews affects consumers’ behavioural responses: the moderating role of dialecticism ✩. *J. Hosp. Tour. Manag.* 41 28–40. 10.1016/j.jhtm.2019.09.003

[B11] AkhtarN.SunJ.ChenJ.Na AkhtarM. (2019b). The role of attitude ambivalence in conflicting online hotel reviews. *J. Hosp. Market. Manag.* 29 471–502. 10.1080/19368623.2019.1650684

[B12] AkramS.NazamM.MubeenR.ChS. R. (2017). Factors influencing effec-tiveness of celebrity endorsement in advertising. *Br. J. Market. Stud.* 5 1–16.

[B13] AlleeK. D.DoC.SterinM. (2021). Product market competition, disclosure framing, and casting in earnings conference calls. *J. Account. Econ.* 72:101405. 10.1016/j.jacceco.2021.101405

[B14] AltıA.SulaemanJ. (2012). When do high stock returns trigger equity issues? *J. Fin. Econ.* 103 61–87. 10.1016/j.jfineco.2011.08.007

[B15] AmanJ.AbbasJ.LelaU.ShiG. (2021). Religious affiliation, daily spirituals, and private religious factors promote marital commitment among married couples: does religiosity help people amid the COVID-19 Crisis? *Front. Psychol.* 12:657400. 10.3389/fpsyg.2021.657400 34421712PMC8377757

[B16] AmanJ.AbbasJ.MahmoodS.NurunnabiM.BanoS. (2019a). The influence of islamic religiosity on the perceived socio-cultural impact of sustainable tourism development in Pakistan: a structural equation modeling approach. *Sustainability* 11:3039. 10.3390/su11113039

[B17] AmanJ.AbbasJ.NurunnabiM.BanoS. (2019b). The relationship of religiosity and marital satisfaction: the role of religious commitment and practices on marital satisfaction among Pakistani respondents. *Behav. Sci. (Basel)* 9:30. 10.3390/bs9030030 30897729PMC6466571

[B18] AmanJ.AbbasJ.ShiG. (2022). Community wellbeing under China-Pakistan economic corridor: role of social, economic, cultural, and educational factors in improving residents’ quality of life. *Front. Psychol.* 12:816592. 10.3389/fpsyg.2021.816592PMC900467035422725

[B19] AmmannM.OeschD.SchmidM. M. (2013). Product market competition, corporate governance, and firm value: evidence from the EU area. *Eur. Fin. Manag.* 19 452–469. 10.1111/j.1468-036X.2010.00605.x

[B20] AndersenT. G.TodorovV.UbukataM. (2021). Tail risk and return predictability for the Japanese equity market. *J. Econometr.* 222 (1. Pt B) 344–363. 10.1016/j.jeconom.2020.07.005

[B21] AnjumM. N.XiuchunB.AbbasJ.ShuguangZ.McMillanD. (2017). Analyzing predictors of customer satisfaction and assessment of retail banking problems in Pakistan. *Cogent. Bus. Manag.* 4:1338842. 10.1080/23311975.2017.1338842

[B22] AnserM. K.ShafiqueS.UsmanM.AkhtarN.AliM. (2020). Spiritual leadership and organizational citizenship behavior for the environment: an intervening and interactional analysis. *J. Environ. Plan. Manag.* 64 1496–1514. 10.1080/09640568.2020.1832446

[B23] AqeelM.AbbasJ.ShujaK. H.RehnaT.ZiapourA.YousafI. (2020). The influence of illness perception, anxiety and depression disorders on students mental health during COVID-19 Outbreak in Pakistan: a web-based cross-sectional survey. *Int. J. Hum. Rights Healthc.* 14 1–14.

[B24] AzadiN. A.ZiapourA.LebniJ. Y.IrandoostS. F.AbbasJ.ChaboksavarF. (2021). The effect of education based on health belief model on promoting preventive behaviors of hypertensive disease in staff of the Iran University of Medical Sciences. *Arch. Public Health* 79 69. 10.1186/s13690-021-00594-4 33952339PMC8097917

[B25] BathiaD.BourasC.DemirerR.GuptaR. (2020). Cross-border capital flows and return dynamics in emerging stock markets: relative roles of equity and debt flows. *J. Int. Money Finance* 109:102258. 10.1016/j.jimonfin.2020.102258

[B26] BhagatS.BoltonB. (2008). Corporate governance and firm performance. *J. Corp. Finance* 14 257–273.

[B27] BloomN.SadunR.ReenenJ. V. (2010). Does product market competition lead firms to decentralize? *Am. Econ. Rev.* 100 434–438.

[B28] BrownL. D.CaylorM. L. (2009). Corporate governance and firm operating performance. *Rev. Quant. Finance Account.* 32 129–144.

[B29] BrownR.LeeN. (2019). Strapped for cash? Funding for UK high growth SMEs since the global financial crisis. *J. Bus. Res.* 99 37–45. 10.1016/j.jbusres.2019.02.001

[B30] BuneaO.-I.CorbosR.-A.PopescuR.-I. (2019). Influence of some financial indicators on return on equity ratio in the Romanian energy sector–a competitive approach using a DuPont-based analysis. *Energy* 189:116251. 10.1016/j.energy.2019.116251

[B31] CarterM. E.ChoiJ.SedatoleK. L. (2021). The effect of supplier industry competition on pay-for-performance incentive intensity. *J. Account. Econ.* 71:101389. 10.1016/j.jacceco.2021.101389

[B32] Chebolu-SubramanianV.SundarrajR. P. (2021). Essential medicine shortages, procurement process and supplier response: a normative study across Indian states. *Soc. Sci. Med.* 278:113926. 10.1016/j.socscimed.2021.113926 33892243

[B33] CrickJ. M.CrickD. (2020). Coopetition and COVID-19: collaborative business-to-business marketing strategies in a pandemic crisis. *Ind. Market. Manag.* 88 206–213. 10.1016/j.indmarman.2020.05.016

[B34] DabworD. T.IoremberP. T.DanjumaS. Y. (2020). Stock market returns, globalization and economic growth in Nigeria: evidence from volatility and cointegrating analyses. *J. Public Aff.* 2020:e2393. 10.1002/pa.2393

[B35] DiasÁL.ManuelE. C.DutschkeG.PereiraR.PereiraL. (2021). Economic crisis effects on SME dynamic capabilities. *Int. J. Learn. Change* 13 63–80. 10.1504/ijlc.2021.111662

[B36] DuarteF. D.Matias GamaA. P.GulamhussenM. A. (2018). Defaults in bank loans to SMEs during the financial crisis. *Small Bus. Econ.* 51 591–608. 10.1007/s11187-017-9944-9

[B37] EggersF. (2020). Masters of disasters? Challenges and opportunities for SMEs in times of crisis. *J. Bus. Res.* 116 199–208. 10.1016/j.jbusres.2020.05.025 32501306PMC7247971

[B38] FarzamiY.Gregory-AllenR.MolchanovA.SehrishS. (2021). COVID-19 and the liquidity network. *Finance Res. Lett.* 42:101937. 10.1016/j.frl.2021.101937 34903955PMC8656191

[B39] FattahiE.SolhiM.AbbasJ.KasmaeiP.RastaghiS.PouresmaeilM. (2020). Prioritization of needs among students of University of Medical Sciences: a needs assessment. *J. Educ. Health Promot.* 9:57. 10.4103/0445-7706.281641 32489992PMC7255571

[B40] FrankoL. G. (1989). Global corporate competition: who’s winning, who’s losing, and the R&D factor as one reason why. *Strateg. Manag. J.* 10 449–474.

[B41] GeT.AbbasJ.AbbasA.UllahR.SadiqI.ZhangR. (2021). Women’s entrepreneurial contribution to family income: innovative technologies promote females’ entrepreneurship amid COVID-19 crisis. *Front. Psychol.* 12:828040. 10.3389/fpsyg.2022.828040PMC900466835422737

[B42] GiroudX.MuellerH. M. (2010). Does corporate governance matter in competitive industries? *J. Financ. Econ.* 95 312–331.

[B43] GiroudX.MuellerH. M. (2011). Corporate governance, product market competition, and equity prices. *J. Finance* 66 563–600. 10.1111/j.1540-6261.2010.01642.x

[B44] GoshitG. G.IoremberP. T. (2020). Measuring the asymmetric pass-through of monetary policy rate to unemployment in nigeria: evidence from nonlinear ARDL. *Niger. J. Econ. Soc. Stud.* 62 369–387.

[B45] GoshitG. G.JelilovG.IoremberP. T.CelikB.Davd-WayasO. M. (2020). Asymmetric effects of monetary policy shocks on output growth in Nigeria: evidence from nonlinear ARDL and Hatemi-J causality tests. *J. Public Aff.* 2020:e2449. 10.1002/pa.2449

[B46] GubarevaM. (2020). The impact of Covid-19 on liquidity of emerging market bonds. *Finance Res. Lett.* 42:101826. 10.1016/j.frl.2020.101826

[B47] GuglerK.WeichselbaumerM.ZulehnerC. (2020). Employment behavior and the economic crisis: evidence from winners and runners-up in procurement auctions. *J. Public Econ.* 182:104112. 10.1016/j.jpubeco.2019.104112

[B48] GuneyY.LiL.FairchildR. (2011). The relationship between product market competition and capital structure in Chinese listed firms. *Int. Rev. Financ. Anal.* 20 41–51. 10.1016/j.irfa.2010.10.003

[B49] GuoS.ZanB.SunY.ZhangM. (2020). Effects of top managers’ military experience on technological innovation in the transition economies of China. *Technol. Forecast. Soc. Change* 153:119909.

[B50] GuptaV. K.HanS.NandaV.SilveriS. (2018). When crisis knocks, call a powerful CEO (or not): investigating the contingent link between CEO power and firm performance during industry turmoil. *Group Org. Manag.* 43 971–998.

[B51] HanH.QianY. (2020). Did enterprises’ innovation ability increase during the COVID-19 Pandemic? evidence from chinese listed companies. *Asian Econ. Lett.* 1:18072.

[B52] HeH.HarrisL. (2020). The impact of Covid-19 pandemic on corporate social responsibility and marketing philosophy. *J. Bus. Res.* 116 176–182. 10.1016/j.jbusres.2020.05.030 32457556PMC7241379

[B53] HibbertA. M.KangQ.KumarA.MishraS. (2020). Heterogeneous beliefs and return volatility around seasoned equity offerings. *J. Financ. Econ.* 137 571–589. 10.1016/j.jfineco.2020.03.003

[B54] HittM. A.HoskissonR. E.JohnsonR. A.MoeselD. D. (1996). The market for corporate control and firm innovation. *Acad. Manag. J.* 39 1084–1119.

[B55] HowellS. T. (2020). Firm type variation in the cost of risk management. *J. Corp. Finance* 64:101691. 10.1016/j.jcorpfin.2020.101691

[B56] HuangM.LiM.LiaoZ. (2021). Do politically connected CEOs promote Chinese listed industrial firms’ green innovation? The mediating role of external governance environments. *J. Clean. Prod.* 278:123634. 10.1016/j.jclepro.2020.123634

[B57] HussainS. T.AbbasJ.LeiS.HaiderM. J.AkramT. (2017). Transactional leadership and organizational creativity: examining the mediating role of knowledge sharing behavior. *Cogent Bus. Manag.* 4:1361663. 10.1080/23311975.2017.1361663

[B58] HussainT.AbbasJ.WeiZ.AhmadS.XuehaoB.GaoliZ. (2021). Impact of urban village disamenity on neighboring residential properties: empirical evidence from nanjing through hedonic pricing model appraisal. *J. Urban Plan. Dev.* 147:04020055. 10.1061/(asce)up.1943-5444.0000645 29515898

[B59] HussainT.AbbasJ.WeiZ.NurunnabiM. (2019). The effect of sustainable urban planning and slum disamenity on the value of neighboring residential property: application of the hedonic pricing model in rent price appraisal. *Sustainability* 11:1144. 10.3390/su11041144

[B60] HutchinsonM.GulF. A. (2004). Investment opportunity set, corporate governance practices and firm performance. *J. Corp. Finance* 10 595–614. 10.1016/S0929-1199(03)00022-1

[B61] IJERPH Editorial Office (2021). Acknowledgments to reviewers of IJERPH in 2020. *Int. J. Environ. Res. Public Health* 18:1259. 10.3390/ijerph18031259

[B62] IlinovaA.DmitrievaD.KraslawskiA. (2021). Influence of COVID-19 pandemic on fertilizer companies: the role of competitive advantages. *Resourc. Policy* 71:102019.10.1016/j.resourpol.2021.102019PMC975968536569185

[B63] IllowskyB.DeanS. (2017). *Introductory Statistics.* Thames Ditton: Samurai Media Limited.

[B64] IoremberP.UsmanO.JelilovG. (2019). *Asymmetric Effects of Renewable Energy Consumption, Trade Openness and Economic Growth on Environmental Quality in Nigeria and South Africa.* Germany: University Library of Munich.

[B65] IoremberP. T.GoshitG. G.DabworD. T. (2020). Testing the nexus between renewable energy consumption and environmental quality in Nigeria: the role of broad-based financial development. *Afr. Dev. Rev.* 32 163–175. 10.1111/1467-8268.12425

[B66] IoremberP. T.JelilovG.UsmanO.IsikA.CelikB. (2021). The influence of renewable energy use, human capital, and trade on environmental quality in South Africa: multiple structural breaks cointegration approach. *Environ. Sci. Pollut. Res. Int.* 28 13162–13174. 10.1007/s11356-020-11370-2 33179189

[B67] IslamT.PitafiA. H.AkhtarN.XiaobeiL. (2021a). Determinants of purchase luxury counterfeit products in social commerce: the mediating role of compulsive internet use. *J. Retail. Consum. Serv.* 62:102596. 10.1016/j.jretconser.2021.102596

[B68] IslamT.PitafiA. H.AryaV.WangY.AkhtarN.MubarikS. (2021b). Panic buying in the COVID-19 pandemic: a multi-country examination. *J. Retail. Consum. Serv.* 59:102357. 10.1016/j.jretconser.2020.102357

[B69] JanuszewskiS. I.KökeJ.WinterJ. K. (2002). Product market competition, corporate governance and firm performance: an empirical analysis for Germany. *Res. Econ.* 56 299–332. 10.1006/reec.2001.0278

[B70] JaveedS. A.LatiefR.LefenL. (2020). An analysis of relationship between environmental regulations and firm performance with moderating effects of product market competition: Empirical evidence from Pakistan. *J. Clean. Prod.* 254:120197. 10.1016/j.jclepro.2020.120197

[B71] JelilovG.IoremberP. T.UsmanO.YuaP. M. (2020). Testing the nexus between stock market returns and inflation in Nigeria: does the effect of COVID-19 pandemic matter? *J. Public Aff.* 20:e2289. 10.1002/pa.2289 32837326PMC7435360

[B72] KhanN.AliK.KiranA.MubeenR.KhanZ.AliN. (2017). Factors that affect the derivatives usage of non-financial listed firms of pakistan to hedge foreign exchange exposure. *J. Bank. Financ. Dyn.* 1 9–20.

[B73] KingM. R.SantorE. (2008). Family values: ownership structure, performance and capital structure of Canadian firms. *J. Bank. Finance* 32 2423–2432. 10.1016/j.jbankfin.2008.02.002

[B74] KoH.-C. A.TongY. J.ZhangF. F.ZhengG. (2016). Corporate governance, product market competition and managerial incentives: evidence from four Pacific basin countries. *Pac. Basin Finance J.* 40 491–502.

[B75] KvalsethT. O. (2018). Relationship between concentration ratio and Herfindahl-Hirschman index: a re-examination based on majorization theory. *Heliyon* 4:e00846. 10.1016/j.heliyon.2018.e00846 30338305PMC6190613

[B76] LebniJ. Y.ToghroliR.AbbasJ.KianipourN.NeJhaddadgarN.SalahshoorM. R. (2021). Nurses’ work-related quality of life and its influencing demographic factors at a public hospital in western iran: a cross-sectional study. *Int. Q. Commun. Health Educ.* 42 37–45. 10.1177/0272684X20972838 33201756

[B77] LebniJ. Y.ToghroliR.AbbasJ.NeJhaddadgarN.SalahshoorM. R.MansourianM. (2020). A study of internet addiction and its effects on mental health: a study based on Iranian university students. *J. Educ. Health Promot.* 9:205. 10.4103/jehp.jehp_148_2033062738PMC7530416

[B78] LeeS.ChangS. R.SuhY. (2020). Developing concentration index of industrial and occupational accidents: the case of european countries. *Saf. Health Work* 11 266–274. 10.1016/j.shaw.2020.05.003 32995052PMC7502666

[B79] LiG.LiJ. (2018). Managerial diversion, product market competition, and firm performance. *China Econ. Rev.* 50 240–264. 10.1016/j.chieco.2018.04.009

[B80] LiM.LuY.PhillipsG. M. (2018). CEOs and the product market: when are powerful CEOs beneficial? *J. Financ. Q. Anal.* 54 2295–2326. 10.1017/S0022109018001138

[B81] LiZ.WangD.AbbasJ.HassanS.MubeenR. (2022). Tourists’ health risk threats amid COVID-19 era: role of technology innovation, Transformation, and recovery implications for sustainable tourism. *Front. Psychol.* 12:769175. 10.3389/fpsyg.2021.769175PMC902277535465147

[B82] LisboaI. (2017). Capital structure of exporter SMEs during the financial crisis: evidence from Portugal. *Eur. J. Manag. Stud.* 22 25–49.

[B83] Liston-HeyesC.PilkingtonA. (2004). Inventive concentration in the production of green technology: a comparative analysis of fuel cell patents. *Sci. Public Policy* 31 15–25. 10.3152/147154304781780190 12543544

[B84] Local Burden of Disease HIV Collaborators (2021). Mapping subnational HIV mortality in six latin American countries with incomplete vital registration systems. *BMC Med.* 19:4. 10.1186/s12916-020-01876-4 33413343PMC7791645

[B85] MahmoodF.HanD.AliN.MubeenR.ShahzadU. (2019). Moderating effects of firm size and leverage on the working capital finance–profitability relationship: evidence from China. *Sustainability* 11:2029.

[B86] MamirkulovaG.MiJ.AbbasJ. (2022). Economic corridor and tourism sustainability amid unpredictable COVID-19 challenges: assessing community well-being in the World Heritage Sites. *Front. Psychol.* 12:797568. 10.3389/fpsyg.2022.797568

[B87] MamirkulovaG.MiJ.AbbasJ.MahmoodS.MubeenR.ZiapourA. (2020). New silk road infrastructure opportunities in developing tourism environment for residents better quality of life. *Glob. Ecol. Conserv.* 24:e01194. 10.1016/j.gecco.2020.e01194

[B88] MaqsoodA.AbbasJ.RehmanG.MubeenR. (2021). The paradigm shift for educational system continuance in the advent of COVID-19 pandemic: mental health challenges and reflections. *Curr. Res. Behav. Sci.* 2:100011. 10.1016/j.crbeha.2020.100011PMC783265438620741

[B89] MeutiaM.IsmailT.UmmiN. (2018). Leadership issue and SME performance during crisis. *Int. J. Civil Eng. Technol.* 9 424–435.

[B90] MichaelidesP. G.TsionasE. G.KonstantakisK. N.XidonasP. (2019). The impact of market competition on CEO salary in the US energy sector1. *Energy Policy* 132 32–37.

[B91] MnasriK.EllouzeD. (2015). Ownership structure, product market competition and productivity. *Manag. Decis.* 53 1771–1805. 10.1108/md-10-2014-0618

[B92] MoradiF.TouraniS.ZiapourA.AbbasJ.HemattiM.MoghadamE. J. (2020). Emotional intelligence and quality of life in elderly diabetic patients. *Int. Q. Commun. Health Educ.* 42 15–20. 10.1177/0272684X20965811 33086936

[B93] MubeenR.HanD.AbbasJ.Alvarez-OteroS.SialM. S. (2021a). The relationship between CEO duality and business firms’ performance: the moderating role of firm size and corporate social responsibility. *Front. Psychol.* 12:669715. 10.3389/fpsyg.2021.669715 35035363PMC8757377

[B94] MubeenR.HanD.AbbasJ.HussainI. (2020). The effects of market competition, capital structure, and CEO duality on firm performance: a mediation analysis by incorporating the GMM model technique. *Sustainability* 12:3480. 10.3390/su12083480

[B95] MubeenR.HanD.AbbasJ.RazaS. (2021b). Examining the relationship between product market competition and Chinese firms performance: the mediating impact of capital structure and moderating influence of firm size. *Front. Psychol.* 12:709678. 10.3389/fpsyg.2021.709678PMC915695635662855

[B96] MubeenR.NazamM.BatoolA.RiazM. (2016). The determinants of capital structure: a case from sugar industry of Pakistan. *Int. J. Manag. Sci. Bus. Res.* 5:191.

[B97] Nasifoglu ElidemirS.OzturenA.BayighomogS. W. (2020). Innovative behaviors, employee creativity, and sustainable competitive advantage: a moderated mediation. *Sustainability* 12:3295. 10.3390/su12083295

[B98] NeJhaddadgarN.ZiapourA.AbbasJ.MardiA.ZareM. (2020a). Correlation between general health and sexual function in older women in an Iranian setting. *J. Educ. Health Promot.* 9:300. 10.4103/jehp.jehp_316_2033426104PMC7774623

[B99] NeJhaddadgarN.ZiapourA.ZakkipourG.AbbasJ.AbolfathiM.ShabaniM. (2020b). Effectiveness of telephone-based screening and triage during COVID-19 outbreak in the promoted primary healthcare system: a case study in Ardabil province, Iran. *Z. Gesundh. Wiss* 29 1–6. 10.1007/s10389-020-01407-8 33224715PMC7665795

[B100] NickellS. J. (1996). Competition and corporate performance. *J. Polit. Econ.* 104 724–746. 10.1086/262040

[B101] PantM.PattanayakM. (2010). Corporate governance, competition and firm performance:evidence from India. *J. Emer. Market Finance* 9 347–381. 10.1177/097265271000900305

[B102] PantanoE.PizziG.ScarpiD.DennisC. (2020). Competing during a pandemic? Retailers’ ups and downs during the COVID-19 outbreak. *J. Bus. Res.* 116 209–213. 10.1016/j.jbusres.2020.05.036 32501307PMC7241368

[B103] PorterM.Van der LindeC. (1995). “Green and competitive: ending the stalemate,” in *The Dynamics of the Eco-Efficient Economy: Environmental Regulation and Competitive Advantage*, ed. WubbenE. F. M. (Cheltenham: Edward Elgar Publishing), 33.

[B104] PouresmaeilM.AbbasJ.SolhiM.ZiapourA.FattahiE. (2019). Prioritizing health promotion lifestyle domains in students of Qazvin University of Medical Sciences from the students and professors’ perspective. *J. Educ. Health Promot.* 8:228. 10.4103/jehp.jehp_250_1931867392PMC6905280

[B105] RahmanM.SaifuzzamanM.AhmedA.MahinM. F.ShetuS. F. (2021). Impact of COVID-19 on mental health: a quantitative analysis of anxiety and depression based on regular life and internet use. *Curr. Res. Behav. Sci.* 2:100037. 10.1016/j.crbeha.2021.100037PMC869084538620872

[B106] RaithM. (2003). Competition, risk, and managerial incentives. *Am. Econ. Rev.* 93 1425–1436.

[B107] Raza AbbasiK.HussainK.AbbasJ.AdedoyinF FataiShaikhP AhmedYousafH. (2021). Analyzing the role of industrial sector’s electricity consumption, prices, and GDP: a modified empirical evidence from Pakistan. *AIMS Energy* 9 29–49. 10.3934/energy.2021003

[B108] Ruiz-PorrasA.Lopez-MateoC. (2011). *Corporate Governance, Market Competition and Investment Decisions in Mexican Manufacturing Firms.* Mexico: Universidad de Guadalajara.

[B109] SaifuzzamanM.RahmanM.Farjana ShetuS.Nessa MoonN. (2021). COVID-19 and Bangladesh: situation report, comparative analysis, and case study. *Curr. Res. Behav. Sci.* 2:100034. 10.1016/j.crbeha.2021.100034PMC805549938620744

[B110] SarfrazR.AqeelM.LactaoJ.KhanS.AbbasJ. (2021). Coping strategies, pain severity, pain anxiety, depression, positive and negative affect in osteoarthritis patients; a mediating and moderating model. *Nat. Nurt. J. Psychol.* 1 18–28.

[B111] ScheidgenK.Aslan GümüsayA.ünzel-JensenF. G.KrlevG.WolfM. (2021). Crises and entrepreneurial opportunities: digital social innovation in response to physical distancing. *J. Bus. Ventur. Insights* 15:e00222.

[B112] SeetharamanP. (2020). Business models shifts: impact of Covid-19. *Int. J. Inf. Manage.* 54:102173. 10.1016/j.ijinfomgt.2020.102173 32834338PMC7323683

[B113] SheikhS. (2018). CEO power, product market competition and firm value. *Res. Int. Bus. Finance* 46 373–386.

[B115] SiddiqiU. I.SunJ.AkhtarN. (2019). The role of conflicting online reviews in consumers’ attitude ambivalence. *Serv. Ind. J.* 40 1003–1030. 10.1080/02642069.2019.1684905

[B116] SiddiqiU. I.SunJ.AkhtarN. (2020). Ulterior motives in peer and expert supplementary online reviews and consumers’ perceived deception. *Asia Pac. J. Market. Logist.* 33 73–98. 10.1108/apjml-06-2019-0399

[B117] SinghS.TabassumN.DarwishT. K.BatsakisG. (2018). Corporate governance and Tobin’s Q as a measure of organizational performance. *Br. J. Manag.* 29 171–190.

[B118] SoininenJ.PuumalainenK.SjögrénH.SyrjäP. (2012). The impact of global economic crisis on SMEs. *Manag. Res. Rev.* 35 927–944. 10.1108/01409171211272660

[B119] SuZ.McDonnellD.AbbasJ.ShiL.CaiY.YangL. (2021a). Secondhand smoke exposure of expectant mothers in china: factoring in the role of culture in data collection. *JMIR Cancer* 7:e24984. 10.2196/24984 34617907PMC8532012

[B120] SuZ.McDonnellD.CheshmehzangiA.AbbasJ.LiX.CaiY. (2021b). The promise and perils of Unit 731 data to advance COVID-19 research. *BMJ Glob. Health* 6:e004772. 10.1136/bmjgh-2020-004772 34016575PMC8141376

[B121] SuZ.McDonnellD.LiX.BennettB.SegaloS.AbbasJ. (2021c). COVID-19 vaccine donations-vaccine empathy or vaccine diplomacy? A narrative literature review. *Vaccines* 9:1024. 10.3390/vaccines9091024 34579261PMC8470866

[B122] SuZ.McDonnellD.WenJ.KozakM.AbbasJ.SegaloS. (2021d). Mental health consequences of COVID-19 media coverage: the need for effective crisis communication practices. *Global. Health* 17:4. 10.1186/s12992-020-00654-4 33402169PMC7784222

[B123] SuZ.WenJ.AbbasJ.McDonnellD.CheshmehzangiA.LiX. (2020). A race for a better understanding of COVID-19 vaccine non-adopters. *Brain Behav. Immun. Health* 9:100159. 10.1016/j.bbih.2020.100159 33052327PMC7544597

[B124] TianG. Y.TwiteG. (2011). Corporate governance, external market discipline and firm productivity. *J. Corp. Finance* 17 403–417.

[B125] ToqeerS.AqeelM.ShujaK. H.BibiA.AbbasJ. (2021). Attachment styles, facebook addiction, dissociation and alexithymia in university students; a mediational model. *Nat. Nurt. J. Psychol.* 1 28–37.

[B126] UsmanO.IOlanipekunO.IoremberP. T.Abu-GoodmanM. (2020). Modelling environmental degradation in South Africa: the effects of energy consumption, democracy, and globalization using innovation accounting tests. *Environ. Sci. Pollut. Res. Int.* 27 8334–8349. 10.1007/s11356-019-06687-6 31900782

[B127] UsmanO.IoremberP. T.OlanipekunI. O. (2019). Revisiting the environmental Kuznets curve (EKC) hypothesis in India: the effects of energy consumption and democracy. *Environ. Sci. Pollut. Res. Int.* 26 13390–13400. 10.1007/s11356-019-04696-z 30905016

[B128] Van ReenenJ. (2011). Does competition raise productivity through improving management quality? *Int. J. Ind. Org.* 29 306–316.

[B129] WangY.HongA.LiX.GaoJ. (2020). Marketing innovations during a global crisis: a study of China firms’ response to COVID-19. *J. Bus. Res.* 116 214–220. 10.1016/j.jbusres.2020.05.029 32501308PMC7247497

[B130] Won Henny JungH.SubramanianA. (2021). Search, product market competition and CEO pay. *J. Corp. Finance* 69:101981. 10.1016/j.jcorpfin.2021.101981

[B131] YangZ.ChenY.ZhangP. (2020). Macroeconomic shock, financial risk transmission and governance response to major public emergencies. *Manag. World* 36 13–35.

[B132] Yoosefi LebniJ.AbbasJ.KhoramiF.KhosraviB.JalaliA.ZiapourA. (2020). Challenges facing women survivors of self-immolation in the kurdish regions of iran: a qualitative study. *Front. Psychiatry* 11:778. 10.3389/fpsyt.2020.00778 32922314PMC7456816

[B133] Yoosefi LebniJ.AbbasJ.MoradiF.SalahshoorM. R.ChaboksavarF.IrandoostS. F. (2021). How the COVID-19 pandemic effected economic, social, political, and cultural factors: a lesson from Iran. *Int. J. Soc. Psychiatry* 67 298–300. 10.1177/0020764020939984 32615838PMC8107447

[B134] YungK.NguyenT. (2020). Managerial ability, product market competition, and firm behavior. *Int. Rev. Econ. Finance* 70 102–116. 10.1016/j.iref.2020.06.027

[B135] ZarembaA.AharonD. Y.DemirE.KizysR.ZawadkaD. (2021). COVID-19, government policy responses, and stock market liquidity around the world: a note. *Res. Int. Bus. Finance* 56:101359. 10.1016/j.ribaf.2020.101359 33343055PMC7717775

[B136] ZhangF.ZhuL. (2021). Social media strategic capability, organizational unlearning, and disruptive innovation of SMEs: the moderating roles of TMT heterogeneity and environmental dynamism. *J. Bus. Res.* 133 183–193. 10.1016/j.jbusres.2021.04.071

[B137] ZhangW.JexS. M.PengY.WangD. (2017). Exploring the effects of job autonomy on engagement and creativity: the moderating role of performance pressure and learning goal orientation. *J. Bus. Psychol.* 32 235–251. 10.1007/s10869-016-9453-x

[B138] ZhaoJ.ChenX.HaoY. (2018). Monetary policy, government control and capital investment: evidence from China. *China J. Account. Res.* 11 233–254.

[B139] ZhouY.DraghiciA.AbbasJ.MubeenR.BoatcaM. E.SalamM. A. (2022). Social media efficacy in crisis management: effectiveness of non-pharmaceutical interventions to manage COVID-19 challenges. *Front. Psychiatry* 12:626134. 10.3389/fpsyt.2021.62613435197870PMC8859332

[B140] ZouH. L.ZengS. X.LinH.XieX. M. (2015). Top executives’ compensation, industrial competition, and corporate environmental performance. *Manag. Decis.* 53 2036–2059. 10.1108/md-08-2014-0515

